# p28 Bacterial Peptide, as an Anticancer Agent

**DOI:** 10.3389/fonc.2020.01303

**Published:** 2020-08-06

**Authors:** Atieh Yaghoubi, Majid Khazaei, Amir Avan, Seyed Mahdi Hasanian, William C. Cho, Saman Soleimanpour

**Affiliations:** ^1^Antimicrobial Resistance Research Center, Bu-Ali Research Institute, Mashhad University of Medical Sciences, Mashhad, Iran; ^2^Department of Microbiology and Virology, Faculty of Medicine, Mashhad University of Medical Sciences, Mashhad, Iran; ^3^Department of Physiology, Faculty of Medicine, Mashhad University of Medical Sciences, Mashhad, Iran; ^4^Metabolic Syndrome Research Center, Mashhad University of Medical Sciences, Mashhad, Iran; ^5^Student Research Committee, Faculty of Medicine, Mashhad University of Medical Sciences, Mashhad, Iran; ^6^Department of Medical Genetics and Molecular Medicine, Faculty of Medicine, Mashhad University of Medical Sciences, Mashhad, Iran; ^7^Department of Medical Biochemistry, Faculty of Medicine, Mashhad University of Medical, Sciences, Mashhad, Iran; ^8^Department of Clinical Oncology, Queen Elizabeth Hospital, Hong Kong, China

**Keywords:** azurin-p28, bacteriotherapy, bacterial peptide, cancer, *pseudomonas aeruginosa*

## Abstract

Cancer remains a major cause of morbidity and mortality irrespective of the type of conventional chemotherapy. Therefore, there is an urgent need for new and effective anticancer therapeutic agents. Bacterial proteins and their derivative peptides appear as a promising approach for cancer treatment. Several, including an amphipathic, α-helical, 28-amino acid peptide derived from azurin, a 128-amino acid copper-containing redox protein secreted from *Pseudomonas aeruginosa*, show clinical promise in the treatment of adult and pediatric solid tumors. The peptide, p28, is a post-translational, multi-target anticancer agent that preferentially enters a wide variety of solid tumor cells. Mechanistically, after entry, p28 has two major avenues of action. It binds to both wild-type and mutant p53 protein, inhibiting constitutional morphogenic protein 1 (Cop1)-mediated ubiquitination and proteasomal degradation of p53. This results in increased levels of p53, which induce cell-cycle arrest at G2/M and an eventual apoptosis that results in tumor cell shrinkage and death. In addition, p28 also preferentially enters nascent endothelial cells and decreases the phosphorylation of FAK and Akt inhibiting endothelial cell motility and migration. Here, we review the current basic and clinical evidence suggesting the potential of p28 as a cancer therapeutic peptide.

## Introduction

Cancer is the second leading cause of death globally with 9.6 million deaths in 2018 (1, 2). Conventional therapies for cancer include surgery, radiotherapy, and chemotherapy. The latter have limitations and adverse side effects, such as a lack of specific toxicity for tumor cells and formation of multidrug resistance. Thus, new therapeutic agents with high treatment efficacy and lower adverse effects are clearly required (3, 4). Recent studies on novel chemotherapeutic approaches to cancer treatment include the use of bacterial therapy (5–7). William Coley (1909) used bacteria and their metabolites to treat cancer. This consists of a mixture of bacterial culture supernatants of *Serratia marcescens* and *Streptococcus pyogenes*, known as “Coley's toxins,” in about 1,200 patients with unresectable tumors. Regression of numerous tumors was observed with complete regression in 30 cases (8). Microbial infection can induce the production of cytotoxic substances that inhibit tumor growth especially tumor necrosis factor-α (TNF-α) through activation of macrophages and lymphocytes (9, 10). This approach has received new attention over the last decade. Several bacterial strains have been used in cancer therapy. These include live, attenuated, or genetically modified bacteria and bacterial products (including bacterial peptides, bacteriocins, and toxins) (11–13). Bacterial peptides and their metabolites, each with unique features, have been used as an anticancer agent. The important advantages of potentially therapeutic bacterial peptides include their small size, easily modifiable features, and rapid, generally simple synthesis (11). In addition to the potential ability to penetrate into the cell membrane, bacterial peptides can exhibit high specificity and affinity for inhibiting the proliferation of different cancer cell lines (14). Moreover, these peptides have shown minimal drug–drug interaction and do not accumulate in specific organs (e.g., kidney or liver), consequently minimizing their toxic side effects (15, 16).

## About Azurin

Azurin is a 128-amino acid (14-kDa) copper-containing member of the cupredoxin family of redox proteins secreted as a periplasmic protein secreted from *Pseudomonas aeruginosa* (17). Azurin has an extended α-helix protein transduction domain (Leu50–Asp77) and four loop regions in its C-terminal including a CD, EF, FG, and GH loop, whose structure is similar to the antibody variable domains of immunoglobulins (18) (Figure 1). A β-sandwich core and an immunoglobulin fold may allow it to escape the immune response and exert its anticancer action (18, 19). In addition to full-length azurin, one peptide, p28 (Leu50-Asp77), derived from azurin also demonstrates anticancer activity (20). Azurin, unlike cell-penetrating cationic peptides that essentially bind to (cancer and normal) cell membrane glycosaminoglycans, preferentially penetrates cancer cells compared to histogenetically similar normal cells through endocytotic, caveosome-directed, and caveosome-independent pathways that make unique these α-helical peptides (21). After preferentially penetrating cancer cells, azurin inhibits the growth of tumor cells leading to tumor cell shrinkage and death via multiple mechanisms including (i) binding to the DNA-binding domain (DBD) of the tumor-suppressor protein p53 and (ii) anti-proliferative and (iii) pro-apoptotic activity (22). Furthermore, azurin is able to inhibit tumor angiogenesis by non-competitively inhibiting the phosphorylation of vascular endothelial growth factor receptor 2 (VEGFR2), as well as the phosphorylation of downstream VEGFR2 targets FAK (focal adhesion kinase), AKT proteins (protein kinase B), and basic fibroblast growth factor (bFGF) (22). In the present article, the anticancer potential of p28 peptide is highlighted as a promising candid for cancer treatment.

**Figure 1:** Primary structure of azurin (128 aa). p28 sequence (28 aa) is derived from amino acids 50 to 77 (Leu50–Asp77) of azurin (in box). This figure is made with I-TASSER (https://zhanglab.ccmb.med.umich.edu/I-TASSER/).

The significant cytotoxicity of azurin toward human carcinomas, such as melanoma, breast, liver, lung, prostate, ovarian, and colorectal sarcoma as well as fibrosarcoma are well-studied (23, 24). The structure of azurin as a scaffold protein includes an invariant β-sheet sandwich formed by parallel and anti-parallel strands as well as an extended α-helix region situated outside the barrel (Figure 1) that may help exert a cytostatic and cytotoxic effect (25–27). Azurin acts by interfering in several signaling pathways associated with cancer progression. It is able to form complexes with the tumor-suppressor protein p53 and increase the intracellular level of this protein by inhibiting the binding of the E3 ubiquitin ligase COP1 to p53 (28, 29). Azurin also shows a topological similarity to ephrins and has the ability to bind to EphB2-Fc receptor tyrosine kinases with high affinity. It has been reported that the G–H loop region in the C-terminal domain of azurin (aa 96–113) has structural similarity to ephrinB2 at the G–H loop region, which has a role in receptor binding. Additionally, azurin could interfere in autophosphorylation of the tyrosine residue in the kinase domain of EphB2 resulting in the prevention of tumor progression and in cancer growth inhibition (30, 31). One previous study reported that azurin is also able to decrease the signaling of the FAK/Src complex, which mediates the decrease in the expression of P-cadherin at the cellular membrane and represses the growth of breast cancer cells with highly invasive P-cadherin overexpression. In addition to the downregulation of P-cadherin levels, treating these cells with azurin leads to maintaining or even increasing the E-cadherin levels, which is known as a tumor-suppressor cadherin protein (32, 33). Each of these mechanisms of action suggests that azurin causes significant regression of several types of solid tumors (34–36).

In addition to *Pseudomonas aeruginosa*, bacteria, such as *Neisseria meningitidis* are able to produce azurin-like proteins (37, 38). Interestingly, one report suggests that the 128-aa azurin would be able to penetrate into glioblastoma cells, when the N-terminal H.8 epitope of the azurin-like protein (Laz) from *N. meningitidis* is fused with azurin, which increases cytotoxicity and may facilitate crossing of the blood–brain barrier to inhibit glioblastomas. Laz, derived from *N. meningitides*, is very similar to azurin of *P. aeruginosa* has a lapidated epitope called H.8 with 39 amino acids located at its N-terminal. The H.8 epitope is responsible for its attachment to the outer membrane and facilitates crossing of the blood–brain barrier (BBB) (21, 37, 38).

The ability of azurin to act as a cell-penetrating peptide is through a protein transduction domain (PTD). One peptide, p28 (aa 50–77; Leu^50^-Asp^77^) of azurin appears to act as both the PTD and the effective inhibitor of cancer cell proliferation (21). Shorter sequences of p28 synthesized to determine the most economical sequence that rendered p28 and its parent azurin able to act as a cell-penetrating peptide included p18 (Leu^50^-Gly^67^), which contains the α-helix domain is the minimal motif for the (PTD) and has a role in the preferential internalization of azurin into the tumor cells (20, 39, 40). Interestingly, p18b aa 60–77 (Val^60^-Asp^77^) is extremely hydrophilic, contains a short α-helix and partial β-sheet, and may negate preferential entry (20). p12 aa 66–77 (Gly^66^-Asp^77^) of azurin 12 aa in length has no secondary α-helical structure but is hydrophilic, which results in the reduction of selectivity of cell penetration (20) (Figure 1). However, this 10 to 12 aa of the COOH terminal of p28 could be responsible for the anti-proliferative activity of p28 (21). Evidence suggests that the cell penetration of azurin, as well as its derivatives p28 and p18, does not result from membrane disruption (21) (Table 1).

**Table 1:** Characteristics of azurin-derived peptides.

**Derived peptides**	**Length (aa)**	**Sequences**	**Positions in azurin**	**Anticancer activities**	**References**
p12	12	SGLDKDYLKPDD	Gly^66^-Asp^77^	Lacks a secondary α-helical structure, hydrophilic p12 has less efficiency in binding p53 Lack of selective penetration	(20, 41, 42)
p18b	18	VTDGMASGLDK DYLKPDD	Val^60^-Asp^77^	Short α-helix and partial β-sheet, hydrophilic p18b has the ability to bind to p53 Lack of selective penetration	(20, 21, 41)
p18	18	LSTAADMQGVVT DGMASG	Leu^50^-Gly^67^	Minimal motif transduction domain (PTD) α-Helix protein High ability in binding to p53 Rapid and preferential penetration into the cancer cells	(20, 21, 41)
p28	28	LSTAADMQGVVTD GMASGLDKDYLKPDD	Leu^50^-Asp^77^	Contains the COOH-terminal region High ability in binding to p53 It has preferential penetration into several cancer cells	(20, 41, 42)

*aa, amino acid*.

## Anticancer Mechanism of p28

### Selective Entry Into Human Carcinoma Cells

The cell-penetrating peptide, p28, Azurin-p28 (NSC745104), has been described as a tumor-homing peptide that preferentially enters tumor cells (21). There is evidence to suggest that p28 enters tumor and normal cells through a receptor-mediated endocytic process including caveolin-1, the Golgi complex, and ganglioside GM-1 (21, 26, 27). Since p28 preferentially enters tumor cells over mature normal cells, one possibility is that there are an increased number of caveolin(-like) receptors, expressed at higher levels on the surface of cancer cells than the surface of normal cells (21, 43). For example, p28 enters human breast cancer cell lines via caveolin-mediated endocytosis. Caveolae are a subset of lipid rafts characterized by the presence of caveolin-1, a known mediator for tumor progression and resistance to standard treatments. Endocytosis mediated by caveolae and lipid raft occurs at neutral pH, which prevents peptide breakdown by intracellular protease or endonuclease, unlike the endocytosis mediated by clathrin. Moreover, evidence showed that uptake of p28, as well as azurin, is energy-dependent and without the disruption in membrane integrity, independent of membrane-bound glycosaminoglycans, dependent on the cholesterol level of the cell membrane. Furthermore, decreasing the cholesterol density of the plasma membranes results in a reduction in the penetration of p28 into the cells (21). However, p28 can enter into cells through clathrin- and caveolin-independent pathways which are not dependent on membrane-bound glycosaminoglycans (21). Thus, these features show that p28 could be used to preferentially transition other peptides to cancer cells (21) (Figure 2).

**Figure 2:** The action mechanisms of Azurin and Azurin-p28 against cancer cells. Azurin and Azurin-p28 enter the cancer cells through planar- or caveolae-lipid raft and cell-surface receptors. Upon entry, p28 destroys the cancer cells by multiple mechanisms.

### Azurin-p28 Interferes With Cellular Signaling Pathways Associated With Cancer

Evidence demonstrates that the COOH terminal 10–12 aa of p28 is the sequence which has a role in inhibiting cell growth and increasing apoptotic activity. Azurin-p28 is a versatile peptide that interferes with several signaling pathways associated with cancer progression. These include the inhibition of angiogenesis and perhaps more importantly induction of a post-translational increase in p53. P28 inhibits angiogenesis and tumor growth even in p53 null tumors by (i) by preventing angiogenesis via decreasing or inhibiting the activity and phosphorylation of VEGFR-2 tyrosine kinase; (ii) inhibiting FAK, AKT, and PI3K phosphorylation; and (iii) inhibiting the effects of bFGF (FGFR-1) on growth. p28 binds to the DNA-binding domain (DBD) of p53, preventing ubiquitination by COP-1 which results in apoptosis and growth inhibition in tumor cells (Figure 2).

Vascular endothelial growth factor receptor 2 (VEGFR2) is expressed in many carcinomas and lymphomas. It is the main responder to vascular endothelial growth factor signal (VEGF), which results in regulation of endothelial migration and proliferation. Therefore, the VEGF/VEGFR2 pathway is a primary therapeutic target in the anti-angiogenic treatment of many solid tumors (22). Exposure of umbilical vein endothelial cells (HUVEC) to p28 reduced their VEGFR-2 kinase activity in response to VEGFA as well as the downstream phosphorylation of FAK and AKT, altering the intracellular structure of the endothelial cytoskeleton and cell-contact proteins, limiting endothelial cell motility and migration of HUVEC (22). Furthermore, p28 inhibition of basic fibroblast growth factor (bFGF) receptors reduces endothelial cell migration, capillary tube formation, and neoangiogenesis in developing tumors. This is interesting as the expression of bFGF and FGFR1 in non-small-cell lung carcinoma (NSCLC) is associated with tumor growth, invasion, and metastasis, although it is not related to the early stage of carcinoma (44). Moreover, FGFR-1 expression in autonomous glioma is related to the increased cell growth and malignant progression (22, 45).

### Interaction of p28 With p53

p53 is a well-known tumor suppressor through apoptosis, growth inhibition, and transcriptional regulation of downstream target genes. Interestingly, p53 has a very short half-life and its basal concentration is regulated through ubiquitin-mediated pathways (46, 47). Numerous studies demonstrate that azurin and p28 are able to inhibit the binding of COP-1 an E3 ubiquitin ligase to the DBD of p53, post-translationally enhancing p53 levels by decreasing the ubiquitination and proteasomal degradation of p53. MDM2 is well-known as a major E3 ubiquitin ligase that is responsible for regulating the degradation of p53 through binding to the N-terminal transactivation domain (TAD) of p53 (48). Initial modeling and physical studies with azurin suggested that its binding to p53 may prevent MDM2 binding to p53, thus preventing the degradation of p53 (28, 49–52). While evidence suggests that azurin may interact with the TA domain of p53, binding kinetics suggest that the complex formed by azurin and p53-TAD (Kd ~ 7 μM) is much larger than the complex formed by MDM2 and p53-TAD (Kd ~ 34 nM), suggesting that azurin is unable to block the binding of MDM2 to the TA domain of p53 (49, 52, 53). Moreover, p28 does not interfere with the binding of MDM2.

Another negative regulator of p53 is COP1, which overexpresses in different cancers, including breast, ovarian, hepatocellular, and gastric cancer. Like azurin, p28 binds to the DBD of p53 primarily at the L1 loop, a structural domain where COP1 also binds (54). Additional overlaps with COP1-binding sites result in the inhibition of the binding of COP1 to p53 and an increase in the stability as well as level of p53 (54–56). Formation of the p28 and p53 complexes induces the transcription of the proapoptotic genes, such as *Bax* and *Noxa*, which interacts with mitochondria, triggering the release of mitochondrial cytochrome c into the cytosol (57–59). This leads, in part, to activation of a caspase cascade and initiation of an apoptotic process. Moreover, the p28-induced increase in p53 produces a cell-cycle arrest at the G2 to M phase through activating the expression of cell-cycle inhibitors, such as p21 and p27. In addition, p28 is able to increase the level of both wild and mutated types of p53 which, in addition to the G2-M cell-cycle arrest, leads to the selective inhibition of cyclin-dependent kinase 2 (CDK2) and cyclin A expression (41, 60). When the peptides that comprise the PTD of azurin, p18 (aa 50–67), p18b (aa 60–77), p12 (aa 66–77), and p28 (aa 50–77) were bound to the p53 DBD, maximum binding to p53 occurred at amino acids 11–18 of p28 (or amino acids 60–67 of azurin) with the 12 amino acids (p12) of the p28 COOH terminal, showing minimal binding efficiency to p53 (41).

p28 is also able to bind to p63 and p73, which are homologs of p53 (29, 61, 62). The p53 family contains three genes that encode p53, p73, and p63 proteins. All three proteins have structural similarities in three main domains that include the transactivation domain (TA), the DNA-binding domain (DBD), and the oligomerization domain (OD) (63). These proteins are considered transcription factors, and these three domains have a crucial role in the downstream transactivation of target genes. The OD domain has a crucial role in the formation of functional tetramers which bind to DNA through the DBD domain. The TA domain is responsible for the transcriptional activity of the family members (63). The binding of p28 to these individual isomers could also enhance the tumor-suppressive activity via a similar mechanism of post-translational stabilization that changes their ubiquitination. Despite the similarity of these proteins in general structure (including a transactivation domain “TA,” a DBD, and a carboxy-terminal oligomerization domain), each protein has individual activities (62).

p63 has a role in embryonic development, epithelial differentiation, and autosomal dominant disorder and tumor suppression, and also it could be an oncogene, while p73 could activate several target genes that promote neuronal and epidermal differentiation, cell-cycle arrest, and cell death. Furthermore, p63 and p73 have a role in the process of cell-cycle regulation, cell death, apoptosis, and differentiation (64, 65). Intracellular levels of p53-family proteins are also regulated through proteasomal pathways mediated by several E3 ubiquitin ligases. The p73 homolog is regulated via the E3 ligase Pirh2, not by COP1, which is bound to the DBD and C-terminus (aa 123–313) of p73 (66–68). In addition, Pirh2 binds to the DBD of p63, while COP1 does not, suggesting that it may not be an important regulator of p63 (66, 69). Collectively, the results demonstrate that p28 is able to bind and interact with the DNA-binding domain of other members of the p53 family including p63 and p73. Furthermore, it can alter the expression of p63 and p73 independent of the MDM2 and COP1 pathways (66).

### p28 as an Anticancer Agent Transporter and Enhancer

p28 is responsible for the preferential entry of azurin into tumor cells (26). Thus, it probably can be used in designing p28-based targeted drug delivery systems. p28 can be used in conjunction with cargo (e.g., anticancer drug) through a linker and then cleaved by enzymatic hydrolysis or form monovalent complexes with the cargos via interactions with liposomes or nanoparticles, all of which should maintain the anticancer activity of p28 and increase the entry of any cancer-targeted agent (25). However, p28 also enters normal cells with rapid-entry kinetics (21). While it also rapidly dissociates, it certainly may increase a normal cell's exposure to higher levels of a toxic agent(s), producing additional non-specific toxic effects. Recently, p28 in combination, sequentially or concurrently, with either DNA-damaging drugs (e.g., doxorubicin, dacarbazine, temozolomide) or anti-mitotic drugs (paclitaxel and docetaxel) was shown to improve the cytotoxic activity of these drugs in a variety of human cancer cells expressing wild-type or mutated p53 and does so at lower concentrations of these agents. It does so by enhancing cytotoxic activity through the p53/p21/CDK2 pathway (70).

## Anticancer Effect of p28 in Different Human Cancer Models

The selective entry and anticancer activity of p28 were examined in cancer preclinical models (Table 2), as follows.

**Table 2:** Anticancer effect of azurin-p28 on different cancer cells with *in vitro* and *in vivo*.

**Cancer type**	**Cancer cell line**	***In vitro***	***In vivo***	**References**
Breast cancer	MCF7, ZR-75-1, T47D, MDA-MB-157, MDD2, MDA-MB-231	1. Anti-proliferation 2. Growth inhibition 3. p53 activation 4. Cytostatic effect 5. High affinity in binding to p63 and p73	1. Reduction of tumor size 2. Inhibition of tumor growth	(41, 71, 72)
Colon cancer	HCT116, HT29	1. p53 activation 2. Specific entry 3. Growth inhibition	NF	(21, 61)
Melanoma	UISO-Mel-6, UISO-Mel-23, UISO-Mel-29, UISO-Mel-2	1. Decrease in survival 2. Specific internalization 3. Proliferation inhibition 4. High-affinity in binding to p63 and p73 5. p53 activation 6. Cytostatic effect 7. Growth inhibition 8. Cytostatic effect 9. Inhibition of motility, migration, and preferential penetration of HUVEC 10. Inhibition of angiogenesis 11. Inhibition of VEGFR-2, FAK, and Akt	1. Proliferation inhibition 2. Reduction of tumor size 3. Inhibition tumor growth	(22, 61, 66)
Glioblastoma	U87, LN229	1. Increase in intracellular levels of p53 2. Significant cytotoxicity	NF	(61, 70)
Prostate cancer	DU145, LNCaP, PC-3	1. Increase in intracellular levels of p53 and p21 2. Anti-proliferation 3. Cytotoxicity 4. Preferential internalization 5. Growth inhibition	NF	(61, 70)
Ovarian cancer	SK-OV3, ES-2	1. Preferential entry 2. Anti-proliferation	NF	(21, 61)
Fibrosarcoma	HT1080	1. Preferential entry 2. Anti-proliferation	NF	(21, 61)
Leiomyosarcoma	HTB-88	1. Preferential entry 2. Proliferation inhibition	NF	(61)
Osteosarcoma	TE85	1. Preferential entry 2. Growth inhibition	NF	(61)
Pancreatic cancer	MIA-Paca2	1. Preferential entry 2. Proliferation inhibition	NF	(61)
Burkitt's lymphoma	Raji, HEK-293	1. Preferential entry 2. Anti-proliferation	NF	(73)
Neuroblastoma	IMR-32, SK-N-BE2	1. Preferential entry 2. Growth inhibition	NF	(70)
Rhabdomyosarcoma	RD	1. Preferential entry 2. Proliferation inhibition	NF	(61)

*NF, not found; HUVEC, human umbilical vein endothelial cells; VEGF, vascular endothelial growth factor; FAK, focal adhesion kinase*.

### p28 and Breast Cancer

p28 preferentially enters MCF-7, T47D, MDA-MB-231, and ZR-75-1 human breast cancer cells ~2- to 3-fold greater than in MCF-10A (normal) cells, irrespective of hormonal or p53 status, and exerts anti-proliferative activity (41, 74). The anticancer activity of p28 on MCF-7, T47D, MDA-MB-231, and ZR-75-1 human breast cancer cell lines is significant. Exposure of MCF-7 cells to 50 μmol/L of p28 demonstrates that the anti-proliferative effect of this peptide was dose- and time-dependent; i.e., the inhibitory effect of p28 increased with time ~9.3% (24 h), ~29% (48 h), and ~50% (72 h). In addition, the inhibitory effect of p28 on the growth of ZR-75-1 cells was also dose-dependent (16% at 50 μmol/L and 44% at 100 μmol/L after 72 h exposure). Moreover, p28 significantly reduced the tumor size of MCF-7 xenografts in athymic mice after exposure to 10 mg/kg (3.4 μmol/kg) of peptide over the course of a daily 30-days i.p course of treatment (41).

It has been suggested that p28 increases the level of the wild-type and mutated p53 without altering its conformation (28). Intracellular levels of p53 are regulated via a group of ubiquitin E3 ligases that promote ubiquitination and proteasome-dependent degradation of p53. COP1 is a major ubiquitin E3 ligase overexpressed in human breast cancers including MCF-7, MDA-MB-231, and T47D, which degrades p53 (28, 75). It has been demonstrated that p28 can enhance the level of the wild-type and mutated p53 by inhibiting the binding of COP1 to p53 (28).

Additional studies show the inhibitory effect of p28 on human breast cancer cell lines as a chimeric protein. Noei et al. (71) engineered a novel chimeric protein composed of the p28 peptide as a tumor-homing killer peptide and apoptin as a killer peptide and evaluated its cytotoxic activity against the breast cancer cell lines MCF7 and MDA-MB-231 (71). Apoptin is a 13.6-kD protein encoded by the chicken anemia virus which induces apoptosis in malignant and transformed cells (76). The results demonstrate a dose-dependent toxicity of chimeric protein comparison to p28 alone on human breast cancer cells; IC50 38.55 and 43.11 μg/mL on MCF7 and MDA-MB-231 cells, respectively (71). A chimeric p28-NRC-03 antimicrobial peptide has also exhibited a dose-related inhibition of MCF7 and MDA-MB-231 breast cancer cell growth (IC50) values of 1.88 and 1.89 μM on MCF7 and MDA MB-231 cells, respectively (72). NRC-03 is a member of the pleurocidin family of cationic antimicrobial peptides (CAPs) that has cytotoxic activity toward multiple breast cancer cell lines. NRC-03 has anticancer activity by damaging the mitochondrial membrane (77).

### p28 and Colon Cancer

Yamada et al. (61) exposed human colon cancer cells (HCT116 and HT29) to 50 and 100 μM of p28 for 24–72 h. The result demonstrates that p28 binds to the specific motifs within the E3 ligase COP1-binding regions of the p53 DBD, subsequently inhibiting COP1-mediated p53 proteasomal degradation and stabilizing p53 (61). The subsequent increase in p53 levels upregulates the downstream molecules p21 and p27 in wild-type p53 and, at least some, mutated p53 cancer cells, leading to inhibition of cancer cell growth (21).

### p28 and Melanoma

Taylor et al. (21) evaluated the effects of p28 on UISO-Mel-2, 23, 29 human melanoma cell lines. The results demonstrate that the penetration of p28 into UISO-Mel-2 cells is temperature and concentration dependent and does not rely on disruption of the cell membrane (21). The decrease in melanoma survival is concentration dependent (100 and 200 μmol/L of p28 decrease the survival of melanoma cell lines UISO-Mel-23 and 29 by 14 and 22%, respectively and is specific as the same concentration of p18 had no significant effect. The inhibition effect of p28 on cancer cell proliferation is initially through a cytostatic mechanism that inhibits the cell cycle and leads to apoptosis. To date, this latter observation appears to be relevant for all solid tumor cell lines (21). A recent study addressed the intracellular level and stability of p53 in UISO-Mel-23 and UISO-Mel-29 melanoma cell lines exposed to p28 for 24–72 h. This resulted in inhibition of COP1 binding and an increase in the levels of wild-type and mutated p53 without altering its conformation (28).

For the anti-proliferative activity of p28 on Mel-29 and Mel-23 human melanoma, the results show the inhibiting effect of p28 on p53^+^ cancer cells *in vitro* and *in vivo*. For this purpose, the human melanoma including Mel-29 and Mel-23 was exposed to 100 μmol/L of p28 for 72 h, which resulted in the cytostatic effect and inhibition growth of Mel-29 and Mel-23. In an *in vivo* study, the concentration of 10 mg/kg of p28 induced a dose-related proliferation inhibition of Mel-23 xenograft tumors, which was comparable with an IC20 dose of DNA alkylating agent dacarbazine (DTIC). Furthermore, the concentration of 4 mg/kg of p28 i.p daily inhibited the growth of human melanoma (UISO-Mel-2) xenografts containing the wild type of p53 (70). The results suggested that p28 inhibited the motility and migration and preferentially penetrated human umbilical vein endothelial cells (HUVEC) after incubation at 37°C for 0.5–24 h with VEGFA (20 ng/ml) ± p28 (25 μmol/l). VEGFA activation of extracellular matrix (ECM) proteins induces endothelial cells to reorganize the cytoskeletal actin. The main angiogenic impact of VEGFA is primarily mediated by the VEGFR-2 receptor. The binding of VEGFA to the VEGFR-2 results in dimer formation then phosphorylation at particular sites and binding to the special molecules which have a role in the cell signaling events associated with cell migration (78, 79). p28 is able to inhibition of VEGFR-2 kinase activity through co-localization with caveolin-1 and VEGFR-2 in membrane-derived caveolae of HUVEC within 30 min after exposure. Furthermore, p28 (16 mg/kg BW; 5.5 μmol/l) was injected i.p. once daily for 7 days to the UISO-Mel-6 xenografts in athymic mice, which resulted in significant inhibition of tumor growth (22).

### p28 and Glioblastoma

Exposure of wild-type p53 U87 (p53wt) and mutated p53 LN229 (p53mut) glioblastoma lines to 50 and 100 μM p28 for 24–72 h resulted in an increase in the intracellular level of p53wt in glioblastoma U87 and downstream levels of p21 in LN229 glioblastoma (61). Longer-term exposure of U87 (p53wt) and LN229 (p53mut) glioblastoma cell lines to 100 μmol/L for 72 h shows that p28 induces significant cytotoxicity (25–30%) in U87 and LN229 glioblastoma cells. Furthermore, the results suggest that p28 increases the level of p53 and p21 in U87 (p53wt) and LN229 (p53mut) cells while decreasing the level of FoxM1 and CDK2 in both cell lines, resulting in cell-cycle inhibition at the G2–M phase (70). This peptide, in combination with DNA-damaging drugs (doxorubicin, dacarbazine, temozolomide) and anti-mitotic drugs (paclitaxel and docetaxel), increased their cytotoxicity by activating p53wt and p53mut, which subsequently induced the endogenous CDK inhibitor p21. The increase in p21 significantly increased their cytotoxic activity, independent of cancer cell type. Therefore, the potential therapeutic value in targeting the p53/p21/CDK2 pathway in combination with lower doses of chemotherapeutic agents improved anticancer efficacy while reducing toxicity (70).

### p28 and Prostate Cancer

The preferential internalization of p28 into DU145 and LNCaP prostate cancer cells provided the impetus to determine its anti-proliferative effect (21). The exposure of p53-mutated (p53mut) DU145 prostate cancer cells to increasing doses and times (h) of p28 showed that DU-145 cells respond to p28 with a decrease in cell proliferation, an increase in intracellular levels of p53 and p21, and no change in the ubiquitin ligase COP1. Furthermore, p28 decreases the cell proliferation in DU145 cells without any or only a minor (5%) change in the conformation of p53 (61). Exposure of DU145 (p53mut, AR-) and additional prostate cancer cell lines LNCaP (p53wt, AR+) and PC-3 (p53null, AR-), increasing the doses and times of p28, suggests that cytostatic, rather than cytotoxic, activity of p28 on LNCaP and DU145 was time- and dose-dependent, decreasing the proliferation of LNCaP and DU145 cell lines by 18 and 22%, respectively. Furthermore, p28 in combination with doxorubicin or paclitaxel enhanced the cytotoxic effect in LNCaP and DU145 (70).

### p28 and Other Cancer Cell Lines

In addition to the cancer cell lines listed above, the preferential entry and anti-proliferative effect of p28 are exhibited on other human cancer cell lines including ovarian cancer cells (SK-OV3 adenocarcinoma and ES-2 ovarian), fibrosarcoma (HT1080), leiomyosarcoma (HTB-88), osteosarcoma (TE85), and rhabdomyosarcoma (RD); pancreatic cancer (MIA-Paca2); Burkitt's lymphoma cell line (Raji and HEK-293); and neuroblastoma (IMR-32 (p53^wt^), and SK-N-BE2 (p53^mut^) (21, 28, 70, 73).

## Clinical Trials of p28

Recently, two phase I trials were carried out to investigate the safety, tolerability, pharmacokinetics, and activity of Azurin-p28 as an anticancer therapeutic. An initial phase I trial was conducted in 15 stage IV cancer patients with multiple solid tumors, such as melanoma, colon, sarcoma, prostate, and pancreas (80). p28 was administered intravenously three times per week over 4 weeks followed by a 2-weeks rest and was given in five gradually rising doses, starting from 0.83 mg p28 per kg body weight, followed by 1.66, 2.5, 3.33, and 4.16 mg per kg body weight of the patients. The side effects as well as the beneficial effects were noted. Results showed no dose-limiting toxicities, significant adverse events, or immune responses to the peptide, even at the highest concentration of Azurin-p28 (80). Seven patients demonstrated stable disease for 7–61 weeks, three a partial response for 44–125 weeks and one a complete response for 139 weeks (80). A second phase I clinical trial enrolled 18 pediatric patients aged 3–21 years with recurrent or progressive central nervous system tumors. Brain tumors are often highly invasive and difficult to treat, since very few drugs can cross the blood–brain barrier to reach the brain tumors. The results showed negligible toxicity for p28 as well as responses in several of these pediatric brain tumor patients (81), prompting the USFDA to approve Azurin-p28 as an orphan drug for the treatment of brain tumor glioma.

## Conclusion and Future Perspectives

Bacterial peptides have attracted attention as a novel therapeutic strategy in the treatment of cancer, especially in patients who have not benefited from conventional cancer therapies. Azurin p28, as a peptide of bacterial origin, demonstrates the promising features of a multi-target anticancer agent with preferential entry and retention into human cancer cells. Azurin-p28 inhibits tumor cell proliferation by inducing cell-cycle arrest and apoptosis via a post-translational increase in p53 in cancer cells. Conventional therapy has a limited effect on numerous solid tumors, particularly glioblastoma due to the blood–brain barrier (BBB) and the invasive nature of glioblastoma (1). Azurin-p28, as a cell-penetrating peptide, is a promising candidate in the treatment of glioblastoma as it interferes with multiple steps of tumor growth including angiogenesis. Two phase I clinical trials of azurin-p28 confirm the safety and anticancer activity of this bacterial peptide in both adult and pediatric patients with advanced-stage or stage IV disease where conventional cancer chemotherapeutic agents are subject to the acquisition of resistance and non-specific toxicity (80, 81). Thus, we suggest recruiting additional adult and pediatric patients with advanced cancer(s) where Azurin-p28 has proven effective in preclinical and clinical studies.

## Author Contributions

SS and AY performed the conceptualization and writing. MK, WC, SH, and AA reviewed and edited the manuscript. All authors contributed to the article and approved the submitted version.

## Conflict of Interest

The authors declare that the research was conducted in the absence of any commercial or financial relationships that could be construed as a potential conflict of interest.
